The article "Analysis of the Clinical Effects of Sodium Valproate and Levetiracetam in the Treatment of Women with Epilepsy during Pregnancy" was retracted in 2023. Reasons: suspected computer-generated content; unreliable results or conclusions; concerns about the data; concerns about the results or conclusions.

# Analysis of the Clinical Effects of Sodium Valproate and Levetiracetam in the Treatment of Women with Epilepsy during Pregnancy

**DOI:** 10.1155/2021/5962200

**Published:** 2021-09-29

**Authors:** Haiqiong Lv, Xiaoying Zhao, Jian Yu

**Affiliations:** ^1^Department of Neurology, Zhuji Hospital Affiliated to Shaoxing University of Arts and Sciences, Shaoxing 311800, Zhejiang, China; ^2^Department of Pharmacy, Zhuji Maternal and Child Health Hospital, Shaoxing 311800, Zhejiang, China

## Abstract

**Objective:**

To explore the clinical effects of sodium valproate and levetiracetam in the treatment of women with epilepsy during pregnancy.

**Methods:**

The clinical data of 124 women with epilepsy during pregnancy who received monotherapy with antiepileptic drugs (AEDs) in our hospital from September 2017 to January 2020 were retrospectively analyzed. According to the type of medication taken by the patients, they were recorded as the sodium valproate group (the VPA group, *n* = 56) and the levetiracetam group (the LEV group, *n* = 68 cases). The effects and the maternal and infant outcomes after treatment were compared between the two groups. The neuron-specific enolase (NSE), cognitive function-related parameters (brain-derived neurotrophic factor (BDNF) and myelin basic protein (MBP)), and related inflammatory factors (tumor necrosis factor- (TNF-) *α* and interleukin- (IL-) 6) levels were compared between the two groups before and after treatment.

**Results:**

After treatment, the total clinical effective rate of the LEV group was 91.18% higher than that of the VPA group 73.21%, and the frequency and duration of seizures were lower than those of the VPA group (*P* < 0.05). After treatment, the probability of gestational hypertension, depression during pregnancy, low-weight infants, and neonatal deformities in the LEV group was lower than that in the VPA group (*P* < 0.05). After treatment, the levels of NSE, MBP, TNF-*α*, and IL-6 in the two groups decreased, and the levels of BDNF increased, and the LEV group changed significantly compared with the VPA group (*P* < 0.05).

**Conclusion:**

Compared with sodium valproate monotherapy, levetiracetam is more effective in controlling seizures and improving maternal and infant outcomes in women with epilepsy during pregnancy and can effectively regulate their neurological and cognitive functions and reduce the serum inflammation factor level.

## 1. Introduction

Epilepsy is a chronic transient brain dysfunction syndrome caused by the abnormally synchronized discharge of the patients' brain neurons [1]. Patients may present with sudden or recurrent neurological disorders, twitching of the limbs, temporary sensory failure, unconscious behavior, and other symptoms [2, 3]. According to statistics from the World Health Organization, among all epilepsy cases, women of childbearing age account for a larger proportion of epilepsy, about 40%, and in these data, most patients with well-controlled seizures are eager to get pregnant and raise offspring [4]. However, existing data show that compared with women of normal childbearing age, women of childbearing age with epilepsy have lower marriage and fertility rates and have a higher risk of complications during pregnancy and childbirth [5, 6]. On the one hand, due to the influence of the metabolism of antiepileptic drugs (AEDs) during pregnancy and the clear or potential teratogenicity of AEDs to the fetus, it brings difficulties to clinical treatment [7, 8]. On the other hand, with the rich selection of AEDs and the increase in the range of indications (such as pain, migraine, and mood disorders), the number of female patients treated with AEDs during pregnancy has increased significantly [9, 10]. Faced with this situation, clinicians should actively seek countermeasures and choose appropriate AEDs to treat epilepsy during pregnancy, so as to provide a favorable guarantee for the safety of mothers and babies in this group.

Sodium valproate is a traditional broad-spectrum AED, which is effective for the treatment of many types of epilepsy. Compared with the new AEDs of levetiracetam and oxcarbazepine, it has the advantage of low price. However, recent studies have shown that when it is used alone or in combination with other AEDs in patients with epilepsy during pregnancy, it has a higher probability of causing fetal malformations than other AEDs. Levetiracetam is a new type of AEDs. Compared with traditional AEDs and other new AEDs, it has a lower incidence of malformations associated with monotherapy in the fetus. Therefore, in recent years, its application in patients with epilepsy during pregnancy has become increasingly widespread. In this study, we observed the clinical effects and safety of sodium valproate and levetiracetam in the treatment of women with peripregnancy epilepsy. The aim was to explore the effects of the above two monotherapies on epilepsy control, maternal and infant outcomes, neurocognitive function, and body inflammatory level in peripregnancy women with epilepsy. The report is as follows.

## 2. Materials and Methods

### 2.1. General Data

This is a retrospective analysis of the clinical data of 124 women with epilepsy during pregnancy who received AEDs monotherapy in our hospital from September 2017 to January 2020. Case inclusion criteria: met the diagnostic criteria of the International Anti-Epilepsy League [11], 22–38 years old, the patients had a history of epilepsy and had at least one epilepsy symptom during pregnancy, the patient without central nervous system disease or space-occupying disease, the patient who signed the consent form, the patient with complete clinical data, and patients who followed doctor's orders and had good medication compliance. Case exclusion criteria: the patient with allergy to sodium valproate or levetiracetam, the patient with neurological or mental disorders and unable to communicate normally, the patient with severe dysfunction such as the heart, liver, and kidney, the patient with severe underlying diseases or tumors, organ transplants, and the patient with the blood system or immune system diseases. According to the type of medication taken by the patients, they were recorded as the sodium valproate group (the VPA group, *n* = 56) and the levetiracetam group (the LEV group, *n* = 68 cases). There was no statistical difference between the general information in Table 1 between the VPA group and the LEV group, and they were comparable (*P* > 0.05).

### 2.2. Treatment Methods

Both groups of patients received routine antiepileptic care and management during the treatment period, including reasonable diet arrangements, avoiding patients from eating foods that may induce epileptic seizures, and providing psychological counseling interventions for patients to relieve the psychological pressure of patients. On this basis, the VPA group received sodium valproate sustained-release tablets (Sanofi (Hangzhou) Pharmaceutical Co., Ltd., approval number: H20010595, specification: 0.5 g × 30 tablets) monotherapy. Usage and dosage: oral 30 min after meal, 2 times/d, initial dose is 10 mg/kg, increase to 20 mg/kg after 1 week, and maintain treatment. The LEV group received levetiracetam tablets (UCB Pharma S. A., approval number: J20160085, specification: 0.5 g × 30 tablets) monotherapy. The usage and dosage are oral 30 min after meal, 2 times/d, the initial dose is 10 mg/kg, increased by 10 mg/kg every week, so that the patient's drug dose at late pregnancy is controlled at 1800 ± 200 mg/kg.

### 2.3. Observation Indicators

1. Therapeutic effect: the criterion of efficacy was based on the revised scoring standard of the International Anti-Epilepsy League [12]. Among them, no epileptic seizures during treatment and no epileptiform discharge on EEG examination were fully controlled. After treatment, the number of epileptic seizures was reduced by 75% or more, and the EEG examination was markedly improved as markedly effective. After treatment, the frequency of epileptic seizures decreased by 50%–<75% and the improvement of EEG was effective. A reduction of less than 50% in the number of seizures was invalid. Total effective number = fully control number + markedly effective number + effective number. Statistics and comparison of the seizure frequency and seizure duration of the two groups of patients.
2. Maternal and infant outcomes: statistics and comparison of the number of cases of placenta previa, premature delivery, miscarriage, gestational hypertension, and depression during pregnancy between the two groups of patients and statistics and comparison of the two groups of fetal cases of fetal distress, stillbirth, low body mass, and neonatal deformities.
3. Serological indicators: the neuron-specific enolase (NSE), cognitive function-related parameters (brain-derived neurotrophic factor (BDNF) and myelin basic protein (MBP)), and related inflammatory factors (tumor necrosis factor- (TNF-) *α* and interleukin- (IL-) 6) levels were compared between the two groups before and after treatment. Detection method: before and after treatment, 6 mL of venous blood was drawn in the morning, centrifuged at 2800 r/min for 8 min, and the supernatant was separated and placed in a refrigerator at −30°C for testing. The detection was carried out by the enzyme-linked immunosorbent method, and the kit was provided by Epson (Shanghai) Biotechnology Co., Ltd.

### 2.4. Statistical Methods

Data analysis was processed by SPSS 22.0 software. The measurement data were expressed as ($\bar{x}$ ± *s*), and *t*-test analysis was used for comparison. The count data were expressed as (%), and *χ*^2^-test analysis was used for comparison. *P* < 0.05 indicated that the difference was statistically significant.

## 3. Results

### 3.1. Comparison of Efficacy between the VPA Group and LEV Group

After treatment, the total clinical effective rate of the LEV group was 91.18% higher than that of the VPA group 73.21% (*P* < 0.05) (Table 2).

### 3.2. Comparison of the Frequency and Duration of Seizures between the VPA Group and LEV Group

After treatment, the frequency of seizures in the LEV group (1.88 ± 0.25) times/month was less than that in the VPA group (2.41 ± 0.23) times/month, and the duration of seizures in the LEV group (2.84 ± 1.01) minutes/time was less than that in the VPA group (3.96 ± 1.21) minutes/time (*P* < 0.05) (Figure 1).

### 3.3. Comparison of Maternal and Infant Outcomes between the VPA Group and LEV Group

After treatment, the incidence of placenta previa, premature delivery, miscarriage, gestational hypertension, and depression during pregnancy in the VPA group was 12.50% (7/56), 16.07% (9/56), 16.07% (9/56), 26.79% (15/56), and 28.57% (16/56), respectively; the incidence of placenta previa, premature delivery, miscarriage, gestational hypertension, and depression during pregnancy in the LEV group was 7.35% (5/68), 13.24% (9/68), 10.29% (7/68), 11.76% (8/68), and 11.76% (8/68), respectively. The incidence of fetal distress, stillbirth, low body mass, and neonatal deformities in the VPA group was 17.86% (10/56), 0.00% (0/56), 83.93% (47/56), and 26.79% (15/56), respectively; the incidence of fetal distress, stillbirth, low body mass, and neonatal deformities in the LEV group was 8.82% (6/68), 0.00% (0/68), 54.41% (37/68), and 5.88% (4/68), respectively. The probability of gestational hypertension, depression during pregnancy, low-weight infants, and neonatal deformities in the LEV group was lower than that in the VPA group (*P* < 0.05) (Figure 2).

### 3.4. Comparison of Serum Indexes between the VPA Group and LEV Group

Before treatment, the NSE levels of the VPA group and LEV group were 14.68 ± 4.36 and 15.01 ± 4.21 ng/mL, BDNF levels were 20.20 ± 2.18 and 20.18 ± 2.21 pg/mL, MBP levels were 3.62 ± 0.45 and 3.65 ± 0.43 *μ*g/mL, IL-6 levels were 13.12 ± 1.66 and 13.15 ± 1.61 pg/mL, and TNF-*α* levels were 3.39 ± 0.43 and 3.41 ± 0.43 ng/mL, respectively. After treatment, the NSE levels of the VPA group and LEV group were 9.13 ± 2.37 and 7.11 ± 2.25 ng/mL, BDNF levels were 30.24 ± 3.52 and 33.68 ± 3.65 pg/mL, MBP levels were 2.56 ± 0.23 and 1.98 ± 0.20 *μg*/mL, IL-6 levels were 9.42 ± 1.15 and 8.20 ± 1.06 pg/mL, and TNF-*α* levels were 1.96 ± 0.20 and 1.24 ± 0.14 ng/mL, respectively. After treatment, the levels of NSE, MBP, TNF-*α*, and IL-6 in the two groups decreased, and the levels of BDNF increased, and the LEV group changed significantly compared with the VPA group (*P* < 0.05) (Figure 3).

## 4. Discussion

According to incomplete statistics, about 0.3–0.7% of women of childbearing age in the world have epilepsy during pregnancy and 0.3–0.5% of children come from women with epilepsy [13–15]. In all patients with epilepsy during pregnancy, the proportion of patients who choose to receive AEDs monotherapy can be as high as 98.6% [16]. Among them, the commonly used AEDs are traditional AEDs such as sodium valproate, carbamazepine, and new AEDs such as lamotrigine, levetiracetam, and oxcarbazepine. Different AEDs are accompanied by different treatment effects and maternal and infant outcomes. This study analyzed and compared the clinical efficacy and safety of sodium valproate and levetiracetam monotherapy. The results showed that after treatment, the total clinical effective rate of the LEV group was 91.18% higher than that of the VPA group 73.21%. At the same time, the frequency and duration of seizures in the LEV group were less than those in the VPA group. It shows that compared with sodium valproate monotherapy, levetiracetam has a better therapeutic effect and can significantly reduce the frequency and duration of seizures in patients with epilepsy during pregnancy. The results also showed that after treatment, the probability of gestational hypertension, depression during pregnancy, low-weight infants, and neonatal deformities in the LEV group was lower than that in the VPA group. This shows that in addition to effective control of seizures during pregnancy, levetiracetam can also effectively reduce the risk of neonatal deformities and low body mass.

Sodium valproate is the first-line AEDs commonly used in clinical practice. It has the advantages of broad antiepileptic spectrum, relatively cheap price, low concentration of drug required, and long action time. Its mechanism of action is related to the promotion of the high expression of the inhibitory neurotransmitter *γ*-aminobutyric acid in the brain, inhibiting the abnormal discharge of neurons, preventing the influx of calcium ions, and maintaining the stability of neuronal cell membranes [17]. At the same time, it is effective in treating bipolar disorder, and it is also the drug of choice for many patients with partial epileptic seizures and has a wide range of clinical applications. However, with the increasing expansion of the scope of clinical application of sodium valproate, its adverse reactions are gradually exposed. Its common adverse effects on patients include skin allergies, thrombocytopenia, personality changes, memory decline, brain cell hypoxia, and liver damage [18]. The adverse effects on the fetus include major congenital malformations (MCMs) such as heart development malformations, bone malformations, urogenital malformations, cleft palate, and neural tube defects [19]. Therefore, it is classified as D-level in the pregnancy safety level by the US Drug and Food Administration. Research on whether the teratogenic risk of AEDs is related to the type of drug, multidrug therapy, and applied dose has found that when the multidrug combination or drug regimen contains sodium valproate, the probability of fetal MCMs is significantly increased [20]. A study comparing the incidence of MCMs during monotherapy found that the incidence of sodium valproate was the highest at 10.3%, which was much higher than the 2.8% of levetiracetam [21]. In this study, the rates of neonatal deformities treated with sodium valproate and levetiracetam were 26.79% and 5.88%, respectively, slightly higher than the study by Meador et al. [20]. This may be caused by the inclusion of some newborns with small deformities in this sample.

Levetiracetam is a pyrrolidone derivative, which can specifically bind to the central nerve synaptic vesicle protein 2A subunit to inhibit the release of neurotransmitters, block the abnormal discharge of neurons, and ultimately reduce seizures [22]. In addition, compared with traditional AEDs such as sodium valproate, it has better drug metabolism, longer action time, and fewer adverse reactions (less impact on the liver, no cognitive impairment, no risk of weight gain, and low probability of skin rash) and other characteristics [23]. Therefore, in recent years, its application in many types of epilepsy has become increasingly widespread, and its use in patients with epilepsy during pregnancy has gradually increased. According to the latest Chinese guidelines for the management of women with epilepsy during peripregnancy, it is recommended that women of childbearing age should give priority to new AEDs for treatment when preparing for pregnancy, but for patients who have used sodium valproate for antiepileptic therapy during pregnancy, if the seizures are well controlled, the applied dose should be adjusted to a lower range, and when the control is not good, you can try to replace or add new AEDs for treatment. It can be seen from the above that although sodium valproate has the advantages of broad-spectrum antiepileptic, it is not recommended as the first-line treatment option for patients with epilepsy during pregnancy. For such patients, levetiracetam has a higher application value in controlling epilepsy and improving maternal and infant outcomes due to its excellent pharmacological and pharmacokinetic properties.

Epilepsy is mostly caused by the abnormal discharge of brain neurons. Long-term repeated seizures can trigger events such as hippocampal neuron regeneration and other central nervous system damage, which in turn leads to cognitive decline in patients [24]. In addition, the release of inflammatory mediators can also increase the excitability of neurons, so it also plays a key role in promoting epileptic seizures [25]. NSE is a marker of nerve damage, and its serum content is positively correlated with the number of neuronal damage [26]. MBP is an important part of myelin sheath, which can reflect the degree of brain nerve damage; when the central nervous system is damaged, its serum level rises; BDNF can prevent neuronal damage and is of great significance to the growth and survival of neurons, and both are important parameters reflecting the cognitive level of patients with epilepsy [27, 28]. Elevated levels of TNF-*α* can excite neurotransmitters, and elevated levels of IL-6 can change neuronal action potentials. The interaction between the two can excite neurons, cause hippocampal damage, and aggravate epilepsy [29]. After treatment, in this study, the levels of NSE, MBP, TNF-*α*, and IL-6 in the two groups decreased, and the levels of BDNF increased, and the LEV group changed significantly compared with the VPA group. It is suggested that compared with sodium valproate monotherapy, levetiracetam monotherapy is more effective in improving neurocognitive function and serum inflammation levels in women with epilepsy during pregnancy. This once again confirmed the good prospects of levetiracetam in the treatment of women with epilepsy during peripregnancy.

In summary, compared with sodium valproate monotherapy, levetiracetam is more effective in controlling seizures and improving maternal and infant outcomes in women with epilepsy during pregnancy and can effectively regulate their neurological and cognitive functions and reduce the serum inflammation factor level.

## Figures and Tables

**Figure 1:** Comparison of the frequency and duration of seizures between the VPA group and LEV group. ^*∗*^Compared with the VPA group, *P* < 0.05.

**Figure 2:** Comparison of maternal and infant outcomes between the VPA group and LEV group (%). (a) Maternal outcomes. (b) Infant outcomes. The incidence of stillbirth in both groups was 0.00%. ^*∗*^Compared with the VPA group, *P* < 0.05.

**Figure 3:** Comparison of serum indexes between the VPA group and LEV group. (a) NSE level. (b) BDNF level. (c) MBP level. (d) TNF-*α* level. (e) IL-6 level. ^*∗*^Compared with the same group before treatment, *P* < 0.05. ^*#*^Compared with the VPA group after treatment, *P* < 0.05.

**Table 1:** Comparison of general information between the VPA group and LEV group.

Information	VPA group (*n* = 56)	LEV group (*n* = 68)	*t*/*χ*^2^	*P*
Age (years)	28.64 ± 4.75	29.40 ± 4.41	0.922	0.358
Disease course (years)	0.65 ± 0.15	0.68 ± 0.14		
Maternal type (cases)			0.020	0.888
Primiparous	32	39		
Multiparous	24	29		
Epilepsy type (cases)			0.374	0.946
Localized	13	15		
Clonic	17	18		
Generalized tonic	15	21		
Generalized tonic-clonic	11	14		

**Table 2:** Comparison of efficacy between the VPA group and LEV group (*n* (%)).

Group	*n*	Fully control	Markedly effective	Valid	Invalid	Total effective
VPA group	56	6 (10.71)	14 (25.00)	21 (37.50)	15 (26.79)	41 (73.21)
LEV group	68	11 (16.18)	29 (42.65)	22 (32.35)	6 (8.82)	62 (91.18)
*t*						5.343
*P*						0.021

## Data Availability

The data used to support the results of this study are available from the corresponding author upon request.
